# *Syzygium aqueum*: A Polyphenol- Rich Leaf Extract Exhibits Antioxidant, Hepatoprotective, Pain-Killing and Anti-inflammatory Activities in Animal Models

**DOI:** 10.3389/fphar.2018.00566

**Published:** 2018-06-05

**Authors:** Mansour Sobeh, Mona F. Mahmoud, Ganna Petruk, Samar Rezq, Mohamed L. Ashour, Fadia S. Youssef, Assem M. El-Shazly, Daria M. Monti, Ashraf B. Abdel-Naim, Michael Wink

**Affiliations:** ^1^Institute of Pharmacy and Molecular Biotechnology, Heidelberg University, Heidelberg, Germany; ^2^Department of Pharmacology and Toxicology, Faculty of Pharmacy, Zagazig University, Zagazig, Egypt; ^3^Department of Chemical Sciences, University of Naples Federico II, Naples, Italy; ^4^Department of Pharmacognosy, Faculty of Pharmacy, Ain Shams University Abbassia, Cairo, Egypt; ^5^Department of Pharmacognosy, Faculty of Pharmacy, Zagazig University, Zagazig, Egypt; ^6^Department of Pharmacology and Toxicology, Faculty of Pharmacy, King Abdulaziz University, Jeddah, Saudi Arabia

**Keywords:** *Syzygium aqueum*, polyphenols, antioxidant, hepatoprotective, pain-killing, anti-inflammatory

## Abstract

*Syzygium aqueum* is widely used in folk medicine. A polyphenol-rich extract from its leaves demonstrated a plethora of substantial pharmacological properties. The extract showed solid antioxidant properties *in vitro* and protected human keratinocytes (HaCaT cells) against UVA damage. The extract also reduced the elevated levels of ALT, AST, total bilirubin (TB), total cholesterol (TC) and triglycerides (TG) in rats with acute CCl_4_ intoxication. In addition to reducing the high MDA level, the extract noticeably restored GSH and SOD to the normal control levels in liver tissue homogenates and counteracted the deleterious histopathologic changes in liver after CCl_4_ injection. Additionally, the extract exhibited promising anti-inflammatory activities *in vitro* where it inhibited LOX, COX-1, and COX-2 with a higher COX-2 selectivity than that of indomethacin and diclofenac and reduced the extent of lysis of erythrocytes upon incubation with hypotonic buffer solution. *S. aqueum* extract also markedly reduced leukocyte numbers with similar activities to diclofenac in rats challenged with carrageenan. Additionally, administration of the extract abolished writhes induced by acetic acid in mice and prolonged the response latency in hot plate test. Meanwhile, the identified polyphenolics from the extract showed a certain affinity for the active pockets of 5-lipoxygenase (5-LOX), cyclooxygenase-1 (COX-1) and cyclooxygenase-2 (COX-2) explaining the observed anti-inflammatory activities. Finally, 87 secondary metabolites (mostly phenolics) were tentatively identified in the extract based on LC-MS/MS analyses. *Syzygium aqueum* displays good protection against oxidative stress, free radicals, and could be a good candidate for treating oxidative stress related diseases.

## Introduction

Reactive oxygen species (ROS) are natural molecules in the body. ROS are formed by the immune system and through mitochondrial oxidative metabolism (aerobic respiration). Environmental stress through drugs, bacterial invasion, heat, heavy metal ions, and exposure to radiation and UV can strongly enhance ROS production (Finkel and Holbrook, 2000).

Reactive oxygen species and/or oxidative stress are able to cause damage to lipids, proteins, and DNA. At the DNA level, ROS can cause mutations of genes that can lead to malfunction of enzymes or regulatory proteins. Thus, ROS can be involved in the pathophysiology of several disorders, including cardiovascular diseases, hypertension, inflammation, cancer and neurodegenerative diseases such as Alzheimer’s and Parkinson’s disease (van Wyk and Wink, 2015, 2017).

Elevated levels of ROS are involved in a number of physiological processes within the human body. Further to wound debridement, they also act as a fundamental host defense compounds and mediators of intracellular signaling cascade. ROS levels in the body are controlled by antioxidative molecules (glutathione) or enzymes (SOD, catalase). A functional interplay between ROS and antioxidants is essential in maintaining cell functions. However, ROS levels can be regulated by the uptake of exogenous antioxidants, among them natural antioxidant secondary metabolites, such as polyphenols, flavonoids, carotenoids, ascorbic acid, or allicin (van Wyk and Wink, 2015, 2017).

Several species belonging to the genus *Syzygium* have been extensively studied for their phytoconstituents as well as their biological activities; among them, *S. cumini*, *S. samarangense*, and *S. jambos*. The reported pharmacological activities include antioxidant, antiviral, anti-diabetic and hepatoprotective properties (Sobeh et al., 2018a,b).

The Water rose apple, *Syzygium aqueum*, a member of family Myrtaceae, is native to Indonesia and Malaysia but is presently widely distributed in the tropics. Several biologically active compounds have been isolated from the plant, among them, epigallocatechin, epigallocatechin gallate, vescalagin, castalagin, and samarangenins A and B (Nonaka et al., 1992). Several plant parts have been used in folk medicine. Substantial anti-hyperglycaemic activities were reported from the leaf extract and its individual components myricitrin, myrilgalone G and B, phloretin and europetin 3-*O*-rhamnoside from plants grown in Malaysia (Manaharan et al., 2012).

In this study, we investigated a methanol extract from *S. aqueum* leaves for its antioxidant activities *in vitro* and in keratinocytes (HaCaT cells). Also, the hepatoprotective activities were studied in a rat model against CCl_4_-intoxicaton; in addition, the anti-inflammatory and antinociceptive activities were analyzed in rat and mouse models. Finally, the active secondary metabolites were characterized using HR-UPLC-MS/MS.

## Materials and Methods

### Plant Material and Extraction

The leaves of *S. aqueum* were collected from trees grown in private garden, Egypt. The species was identified by Mrs. Therese Labib, Consultant of Plant Taxonomy at the Ministry of Agriculture and El-Orman Botanical Garden, Giza, Egypt. A voucher specimen (accession number: PHG-P-SA-181) was deposited at Pharmacognosy Department, Faculty of Pharmacy, Ain Shams University. The air-dried and milled leaf powder (100 g) was extracted with 100% methanol at ambient temperature (3 × 500 mL). The whole mixture was filtered and concentrated under vacuum at 40°C giving a semisolid residue. The latter was frozen at -70°C and lyophilized for 72 h yielding fine dried powder (12 g).

### LC–HRESI-MS–MS

An HPLC Agilent 1200 series instrument was used to analyze the sample. A Gemini 3 μm C18 110 A° column from Phenomenex with dimensions 100 × 1 mm i.d., protected with RP C18 100 A° guard column with dimensions (5 mm × 300 μm i.d., 5 μm) was used. The mobile phase was (A) 2% acetic acid and (B) 90% MeOH, 2% acetic acid at a flow rate of 50 μL/min. The gradient was from 5% B at 0 min to 50% B in 50 min and then increased to 90% in 10 min and kept for 5 min. Fourier transform ion cyclotron resonance mass analyzer was used equipped with an electrospray ionization (ESI) system. The system was controlled using X-calibur^®^ software. The data were collected in the negative ion mode as described before (Sobeh et al., 2018b). The full mass scan covered the mass range from 150 to 2000 *m/z* with resolution up to 100000.

### Biological Activity

#### Antioxidant Activities *in Vitro*

Total phenolic contents were determined using the Folin-Ciocalteu method and the antioxidant activities were investigated by DPPH radical scavenging activity, FRAP assay and ABTS assay, as previously described (Ghareeb et al., 2017).

#### Total Antioxidant Capacity (TAC) Assay

Total antioxidant capacity was assessed using a commercially available TAC ELISA kit (MBS726896, MyBioSource, Inc., San Diego, CA, United States) according to the manufacturer’s instructions using ascorbic acid as the reference standard. Briefly, the extract, ascorbic acid or PBS were incubated with TAC-HRP conjugate in pre-coated plate for 1 h. This was followed by proper washing and incubation with a substrate for HRP enzyme. A yellow color was formed which is inversely proportional to the TAC concentration. After 30 min, the stop solution was added to terminate the reaction. The intensity of the yellow color formed was measured at 450 nm in a microplate reader (Molecular Devices, Sunnyvale, CA, United States). A standard curve was established using serial dilutions of the standard. The sample activity (U/L) was calculated from the standard curve equation.

#### Cell Culture and MTT Assay

Human epidermal keratinocytes (HaCaT), provided by Innoprot (Biscay, Spain), were cultured as described in Petruk et al. (2016). For dose and time dependent biocompatibility experiments, cells were seeded in 96-well plates at a density of 2 × 10^3^cells/well. Twenty four hour after seeding, increasing concentrations of the methanol extract (from 25 to 200 μg/mL) were added to the cells for 24 and 48 h. Cell viability was assessed by the MTT [3-(4,5-dimethylthiazol-2-yl)-2,5-diphenyltetrazolium bromide] assay as described in Monti et al. (2015). Cell survival was expressed as the percentage of viable cells in the presence of the extract compared to controls. Two groups of cells were used as control, i.e., untreated cells and cells supplemented with identical volumes of buffer. Each sample was tested in three independent analyses, each carried out in triplicates.

#### Oxidative Stress in HaCaT Cells

To investigate oxidative stress, HaCaT cells were plated at a density of 2 × 10^4^ cells/cm^2^. Twenty four hour after seeding, cells were incubated for 2 h in the presence or absence of 100 μg/mL of the extract and then exposed to UVA (100 J/cm^2^). Then, ROS levels, intracellular GSH levels and the phosphorylation of p38 were analyzed as described in Petruk et al. (2016). The other assays namely DCFDA assay, DTNB assay and Western blot analyses were performed as described in Petruk et al. (2016).

#### Hepatoprotective Activity *in Vivo*

##### Animals and experimental design

Male Sprague-Dawley rats, weighing 200–250 g, were purchased from the animal resource branch, King Abdulaziz University, Geddah (KSA). The rats were fed on rodent chow and water *ad libitum* and housed in conventional cages at 22 ± 2°C, with a 12 h light–dark cycle. The study protocol was approved by the Unit of Biomedical Ethics Research Committee, Faculty of Medicine, King Abdulaziz University, following the Institutional Animal Care and Use Committee guidelines (Reference # 157-14). In brief, 24 rats were divided into four groups. Group (1) served as a control and obtained water orally followed by intraperitoneal (i.p.) injection of corn oil after 4 h. Group (2) was injected a single dose of CCl_4_-corn oil (Sigma–Aldrich, St. Louis, MO, United States) (1 ml/kg, of 50% mixture). Group (3) served as a positive control and was administered the known hepatoprotective silymarin (200 mg/kg orally). Group (4) was pretreated with *S. aqueum* extract (200 mg/kg orally). Groups (3 and 4) were injected CCl_4_-corn oil (1 ml/kg, of 50% mixture, i.p.) after 4 h from the pretreatment (Sobeh et al., 2018a).

Twenty four hour after the treatments, the rats were anesthetized, and blood samples were collected by cardiac puncture, allowed to clot, centrifuged for 10 min at 2113 ×*g*, and then kept at -80°C until analysis. Finally, the rats were sacrificed, and liver tissues were dissected. The liver tissues were cut and fixed in 10% formalin/saline and embedded in paraffin for histopathological investigations. The remaining liver tissues were re-weighed, washed and homogenized in ice-cold PBS to yield 10% w/v homogenates and then stored at -80°C until analyses.

##### Liver biomarkers

Mindray BS-120 clinical chemistry auto-analyzer (Shenzhen Mindray Bio-Medical Electronics Co. Ltd., Shenzhen, China) was used to determine the activities of alanine aminotransferase (ALT), aspartate aminotransferase (AST), total bilirubin (TB), total cholesterol (TC), and triglycerides (TG). The levels of oxidative stress markers glutathione (GSH), lipid peroxidation marker malondialdehyde (MDA) and the activity of the antioxidant enzyme superoxide dismutase (SOD) were quantified utilizing the commercially available kits (Biodiagnostics, Cairo, Egypt).

##### Histopathological examination

Liver tissue samples were stored in 10% buffered neutral formalin for 24 h and then washed with tap water. Dehydration was conducted using serial dilutions of methyl, ethyl and absolute ethyl alcohols. The tissue sections were then embedded in xylene, immersed in paraffin, and dried inside hot air oven at 56°C for 24 h. Tissue sections, 4 μm thickness, were prepared using slide microtome, placed on glass slides, and stained with eosin and hematoxylin. The latter was investigated using the light electric microscope (Olympus BX-50 Olympus Corporation, Tokyo, Japan) as described in Sobeh et al. (2018a).

#### Anti-inflammatory Activities

##### *In Vitro* Anti-inflammatory activities

The capacity of the extract to inhibit lipoxygenase was determined using a lipoxygenase inhibitor screening assay kit (Cayman Chemical, Ann Arbor, MI, United States) according to the manufacturer’s instruction and reported study (Abdelall et al., 2016). The ability of the extract to inhibit ovine COX-1 and COX-2 was determined by using an enzyme immunoassay (EIA) kit (Cayman Chemical, Ann Arbor, MI, United States) according to the manufacturer’s instruction and reported studies (Abdelall et al., 2016). The data are expressed as IC_50_ value, which is the concentration causing 50% enzyme inhibition (IC_50_). Furthermore, the COX-2 selectivity index (SI values) which is defined as IC_50_ (COX-1)/IC_50_ (COX-2) was calculated and compared to that of celecoxib, indomethacin, and diclofenac which were used as reference standards.

##### Membrane stabilizing activity (hypotonic solution-induced hemolysis)

The membrane stabilizing activity of the extract was assessed in erythrocytes; hemolysis was induced by osmotic shock (Shinde et al., 1999). Fresh whole blood (10 mL) was collected from a healthy human volunteer who had not taken any NSAIDS for 2 weeks prior to the experiment. This was followed by centrifugation of heparinized blood (2113 ×*g*/10 min) and washing with normal saline. Next, a 40% (v/v) RBCs suspension in 10 mM sodium phosphate buffer solution (NaH_2_PO_4_. 2H_2_O, 0.26 g; Na_2_HPO_4_, 1.15 g; NaCl, 9 g) was prepared. A 0.5 mL of the previous suspension was incubated for 10 min with 5 mL of hypotonic solution (50 mM NaCl in 10 mM sodium phosphate buffered saline, pH 7.4) containing with the extract (1000 μg/mL), aspirin or diclofenac (100 μg/mL) as reference drugs. The samples were then centrifuged at 3000 *g* for10 min. The absorbance of the supernatant was then detected at 540 nm. The ability of the tested sample to inhibit RBCs hemolysis was calculated using the following equation:

Hemolysis inhibition %=(ODI−OD2/OD1)×100

where OD1 = Optical Density of the control (cells incubated with the buffer only) and OD2 = Optical Density of test sample.

##### Carrageenan-induced hind-paw edema

Right hind paw edema was induced in rats by injecting freshly prepared carrageenan solution (1% in 0.9% NaCl, 0.1 mL), into the sub plantar tissue. 1 h earlier, the vehicle (10 mL/kg), *S. aqueum* extract (300 mg/kg, p.o.) or diclofenac (10 mg/kg) were given orally. The paw thickness (mm) was measured in the dorsal- plantar axis by a caliper ruler before and after the carrageenan injection at hourly intervals for 6 h and then at 24 h. The cumulative anti-inflammatory effect during the whole observation period (0–24 h) was estimated by calculating the area under changes in paw thickness-time curve (AUC_0-24_).

##### Recruitment of leukocyte to peritoneal cavity in mice

The recruitment of leukocytes to the peritoneal cavity was assessed as described previously (Silva-Comar et al., 2014). Briefly, Swiss albino mice (*n* = 5–8/group), were orally treated with the vehicle (1 mL/100 g, p.o.) or *S. aqueum* extract (300 mg/kg) 30 min before the intraperitoneal injection of 0.1 mL carrageenan solution (500 μg/mice) or 0.1 mL sterile saline. Diclofenac (10 mg/kg, p.o.) was used as the reference anti-inflammatory drug. The animals were euthanized 3 h later and the peritoneal cavity was washed with 3 mL of phosphate-buffered saline (PBS) contained 1 mM ethylenediaminetetraacetic acid (EDTA). The total leukocyte count was determined in the peritoneal cavity wash using a hemocytometer and expressed as number of cells/mL.

#### Antinociceptive Activity

##### Acetic acid-induced abdominal writhing

The peripheral analgesic activity of the extract was evaluated using acetic acid induced writhing model in mice (Nakamura et al., 1986). The animals were divided into three groups (5–7 mice). Group (1) received the vehicle (1% Tween 80, 10 mL/kg) and served as negative control. Group (2) received the extract (300 mg/kg, p.o.) and group (3) received diclofenac (10 mg/kg, a reference drug) 1 h prior i.p. injection of 0.7% acetic acid (1 mL/100g). The number of writhes (constriction of abdomen, turning of trunk and extension of hind legs) was observed for 25 min.

##### Hot plate test

The hot plate test was carried out to test a possible central analgesic activity of the extract (Macdonald et al., 1946; Eddy and Leimbach, 1953). Mice were divided in different groups (5 each) and receive either the extract (300 mg/kg, p.o.) or the vehicle (10 mL/kg, p.o.). Another group of mice received the opioid analgesic nalbuphine as reference central analgesic. After 60 min, the mice were individually placed in a hot plate heated at 55 ± 1°C and the animal was studied for any sign of response to heat-induced nociceptive pain (licking of the fore and hind paws, hind paw lifting or jumping). The latency until mice showed the first signs of discomfort was recorded before (baseline) and at 1, 2, 3, and 4 h following different treatments.

### Molecular Modeling

*In silico* virtual screening studies of the major constituents identified in the bioactive methanol extract of *S. aqueum* was performed using the C-docker protocol on 5-lipoxygenase (PDB ID 3V99, 2.48 Å), cyclooxygenase-I (PDB ID 2OYE, 2.85 Å) and cyclooxygenase-II (PDB ID 3LN1, 2.3 Å) that were downloaded from protein data bank^1^. This was done by applying both pH and rule-based ionization methods for the preparation of ligands with Discovery Studio 2.5 (Accelrys Inc., San Diego, CA, United States). *In silico* virtual screening was performed within the active pocket of the previously mentioned enzymes and the free binding energies for the highly stable docking poses were calculated as previously discussed (Sobeh et al., 2016; Ashour et al., 2017; Youssef et al., 2017).

### Data Analysis

Data were analyzed using GraphPad Prism software, version 5.00 (GraphPad Software, Inc., La Jolla, CA, United States). Analysis of Variance (ANOVA) or repeated-measures analysis of variance (RM-ANOVA) followed by Tukey’s *post hoc* test and Student’s *t*-test were used to state differences between groups. Otherwise mentioned, data are expressed as mean ± SEM.

## Results

### Secondary Metabolites From *S. aqueum*

Utilizing high resolution LC-ESI-MS/MS, 87 compounds were characterized in a methanol extract of *S. aqueum* leaves. Flavonoids, represented by myricetin rhamnoside (**53**), myrigalone-G pentoside (**71**), quercetin galloyl-pentoside (**73**), cryptostrobin (**87**), myrigalone-B (**85**), and myrigalone-G (**86**) dominated the extract, in addition, proanthocyanindins with mainly samarangenin A (**27**), (epi)-gallocatechin gallate (**33**), and (epi)-catechin-(epi)-gallocatechin-(epi)-gallocatechin gallate (**36**) were abundant. Also, digalloyl-hexahydroxydiphenoyl (HHDP)-hexoside (**37**), as an example for ellagitannins, was among the major constituents. Some phenolic acid derivatives and other ellagitannins were characterized as well (**Figure 1** and **Table 1**). Representative MS/MS fragmentation of some identified compounds are presented in Supplementary Figures S1–S45.

**FIGURE 1:** HR-LC-MS/MS chromatogram of a methanol extract from *S. aqueum* leaves.

**Table 1:** Secondary metabolites from a methanol extract of *S. aqueum* leaves by HR-LC-MS/MS.

No.	t_R_(min)	[M-H]^-^	MS/MS fragment	Tentatively identified compounds
1	1.63	191	127	Quinic acid^a^
2	2.23	341	179	Caffeoyl hexoside
3	2.87	343	191	Galloylquinic acid^a^
4	3.02	331	169	Galloyl hexose^a^
5	3.26	609	305, 423, 441, 591	(epi)-Gallocatechin-(epi)-gallocatechin
6	3.88	483	169, 331	Digalloyl hexose
7	4.43	933	301, 301, 631, 915	Castalagin/Vescalagin^∗,a^
8	6.13	477	169, 313, 331	Gallic acid coumaroyl-hexose
9	6.28	633	301, 463, 615	Galloyl-hexahydroxydiphenoyl (HHDP)-hexoside
10	6.36	609	305, 423, 441	(epi)-Gallocatechin-(epi)-gallocatechin^a^
11	6.51	343	125, 169	Galloylquinic acid
12	6.76	1583	765, 935, 1537, 1565	Eugeniflorin D2^a^
13	7.85	305	125, 179	(epi)-Gallocatechin^∗,a^
14	9.14	179	161	Caffeic acid
15	9.27	315	153	*p*-Coumaric acid hexoside
16	10.29	441	179, 271, 423	(epi)-Catechin gallate
17	12.23	301	229, 257, 301	Ellagic acid^b^
18	12.87	593	289, 425, 557	(epi)-Catechin-(epi)-gallocatechin
19	16.12	761	305, 423, 593, 609	(epi)-Gallocatechin-(epi)-gallocatechin gallate^a^
20	17.11	897	305, 559, 609, 771	(epi)-Gallocatechin-(epi)-gallocatechin-(epi)-catechin
21	17.81	783	301, 615, 765	Pedunculagin^∗^
22	18.21	273	187, 229	(epi)-Afzelechin
23	19.90	633	301, 481, 615	Galloyl-hexahydroxydiphenoyl (HHDP)-hexoside
24	21.20	745	289, 577, 593, 727	(epi)-Catechin-(epi)-gallocatechin gallate^a^
25	22.61	285	153	*p*-Coumaric acid pentoside
26	22.72	483	169, 331	Digalloyl hexose
27	23.41	759	229, 301, 633	Samarangenin A^∗^
28	24.79	577	289, 407, 425, 559	(epi)-Catechin-(epi)-catechin^a^
29	25.74	745	305, 423, 457, 593	(epi)-Gallocatechin-(epi)-catechin gallate^a^
30	25.94	575	287, 423	(epi)-Catechin-A-(epi)-catechin
31	28.25	761	305, 423, 609	(epi)-Gallocatechin-(epi)-gallocatechin gallate
32	28.91	785	301, 483, 633, 765	Digalloyl- HHDP-hexoside
33	29.89	457	305, 331	(epi)-Gallocatechin gallate^∗,a,¥^
34	33.48	745	289, 441, 593, 619	(epi)-Gallocatechin-(epi)-catechin gallate^a^
35	33.7	1217	423, 761, 1047, 1065	(epi)-Gallocatechin-(epi)-gallocatechin-(epi)-gallocatechin-(epi)-gallocatechin^a^
36	34.92	1049	423, 745, 761	(epi)-Catechin-(epi)-gallocatechin -(epi)-gallocatechin gallate^a^
37	35.94	785	301, 483, 615, 633, 765	Digalloyl-HHDP-hexoside
38	37.00	1201	423, 475, 1049	(epi)-Catechin-(epi)-gallocatechin-(epi)-gallocatechin-(epi)-gallocatechin
39	37.27	367	191	Feruloylquinic acid
40	37.5	337	191	*p*-Coumaroylquinic acid^a^
41	38.82	881	423, 591, 729	(epi)-catechin gallate-(epi)-catechin gallate
42	40.71	1217	423, 761, 913, 1030	(epi)-Gallocatechin-(epi)-gallocatechin-(epi)-gallocatechin-(epi)-gallocatechin^a^
43	41.09	441	169, 289	(epi)-Catechin gallate^∗,a^
44	42.18	1017	407, 575, 729	(epi)-Catechin-(epi)-catechin-(epi)-catechin gallate^a^
45	42.23	913	423, 591, 761	Prodelphinidin B2 3,3′-digallate^∗^
46	43.13	451	169, 289	(epi)catechin glycoside
47	45.41	911	285, 423, 571, 759	Samarangenin B^∗^
48	49.03	625	317, 463	Myricetin rhamnosyl-hexoside^a^
49	49.53	479	317	Myricetin hexoside^a^
50	50.27	449	179, 317	Myricetin pentoside^a^
51	51.72	595	179, 271, 301, 463	Quercetin pentosyl-hexoside
52	52.08	623	285, 447	Myrigalone-G glucuronide-hexoside
53	53.15	463	179, 317	Myricetin3-*O*- rhamnoside^∗,a,¥^
54	54.43	375	361	Methyligstroside aglycone
55	54.83	631	317, 479	Myricetin galloly-hexoside
56	56.85	729	289, 407, 559	Procyanidin dimer monogallate^a^
57	57.15	593	285, 447	Myrigalone-G rhamnosyl-hexoside
58	57.22	601	317, 449	Myricetin galloyl-pentoside
59	57.9	881	289, 407, 559, 729	(epi)-Catechin gallate-(epi)-catechin gallate^a^
60	58.08	493	331	Europetin hexoside
61	58.18	609	301	Quercetin rutinoside^a^
62	58.33	645	331, 493	Europetin galloly-hexoside
63	58.51	737	300, 433	Quercetin pentosyl digallate
64	58.58	749	301, 447, 595, 597	Quercetin rhamnosyl-digallate
65	62.17	433	301	Quercetin pentoside
66	63.36	477	331	Europetin rhamnoside^∗^
67	63.84	447	301	Quercetin rhamnoside
68	64.04	615	317, 463	Myricetin galloyl-rhamnoside^a,c^
69	64.13	615	301, 463	Quercetin galloyl-hexoside^a^
70	64.8	447	315	Isorhamnetin pentoside
71	64.98	417	285	Myrigalone-G pentoside
72	65.28	461	315	Isorhamnetin rhamnoside
73	65.3	585	301, 433	Quercetin galloyl-pentoside^a^
74	66.34	601	179, 317, 449	Myricetin galloyl-pentoside
75	66.43	935	301, 463, 633, 783	Quercetin hexoside trigallate
76	67.01	599	301, 447	Quercetin galloyl-rhamnoside
77	67.36	615	317, 463	Myricetin galloyl-rhamnoside^a^
78	68.06	417	285	Myrigalone-G pentoside
79	68.15	523	361	Ligstroside
80	68.26	431	285	Myrigalone-G rhamnoside
81	68.27	329	285	Acetylemyrigalone-G^∗^
82	69.09	461	329	Tricin pentoside
83	69.35	585	179, 301, 433	Quercetin galloly-pentoside
84	71.56	629	179, 301, 463, 477	Quercetin methyl galloyl-hexoside
85	72.11	299	151, 243, 271	Myrigalone-B^∗^
86	73.36	285	163, 241, 271	Myrigalone-G^∗^
87	74.20	269	121, 255, 271	Cryptostrobin^a^

*^∗^Previously isolated from the plant (Nonaka et al., 1992) and (Manaharan et al., 2012). ^¥^Identification was confirmed using authentic standard compounds. ^a^Identification was based on Sobeh et al. (2018b). ^b^Identification was based on Sobeh et al. (2018a).*

### Antioxidant Activities *in Vitro* and in Keratinocytes

Initially, we evaluated the antioxidant potential of the leaf extract *in vitro* using DPPH^⋅^, TEAC and FRAP assays as well as total antioxidant capacity (TAC), as reported in **Table 2**. The total phenolic content amounted to 453 mg GAE/g extract. The extract demonstrated substantial activities in all assays. (epi)Gallocatechin gallate (EGCG) and ascorbic acid were used as reference compounds.

**Table 2:** Antioxidant properties of the extract as compared to positive controls EGCG and vitamin C.

Assay	*S. aqueum* extract	EGCG	Ascorbic acid
DPPH (EC_50_ μg/mL)	6.80 ± 0.15	3.50 ± 0.23	2.95 ± 0.13
TEAC (Trolox equivalents/mg of sample)	2073 ± 17	5293 ± 23	-
FRAP (Fe^2+^ equivalents/mg of sample)	11.51 ± 0.82	25.23 ± 1.32	-
TAC (Total antioxidant capacity, U/L)	18.72 ± 1.11		26.41 ± 1.75

We also investigated the antioxidant capacity of the extract in human keratinocytes. First, we tested the biocompatibility of the extract in HaCaT cells by a time-course and dose-response test, using increasing amount of extract (from 25 to 200 μg/mL). As shown in **Figure 2A**, cell viability was not significantly affected at any of the concentration and time analyzed. Then, we investigated whether the extract had protective properties against oxidative stress. In all the experiments, cells were pre-treated with the extract (100 μg/mL) for 2 h before challenging cells with UVA irradiation to induce oxidative stress (100 J/cm^2^). At the end of the incubation, intracellular ROS levels were analyzed by using H_2_DCF-DA (2,7-dichlorofluorescin diacetate) (**Figure 2B**). It is apparent that UVA significantly increased DCF fluorescence intensity, compared to the non-irradiated cells. However, pre-treatment of the cells with the extract showed reduced ROS levels. The UVA induced increase in ROS levels is normally followed by a decrease in total GSH levels. In fact, as shown in **Figure 2C**, cells irradiated by UVA have dramatically reduced GSH levels. As expected, cells pre-treated with the extract and then exposed to oxidative stress showed unaltered GSH levels, compared to the untreated cells. The ability of the extract to protect HaCaT cells from UVA damages was confirmed by Western blot analysis. In particular, a mitogen activated protein kinase (p38) phosphorylation levels were analyzed (**Figure 2D**). We found that treatment of cells with extract does not activate this protein. Instead, as expected, UVA induced a significant increase in the phosphorylation levels of p38. On the other hand, when cells were pre-incubated with the extract and then exposed to UVA radiations, the phosphorylation levels of p38 were significantly lower to that observed in irradiated cells.

**FIGURE 2:** Effect of *Syzygium aqueum* extracts on human keratinocytes. **(A)** Biocompatibility of *S. aqueum* extract in dose (25–200 μg/mL) and time (24–48 h) manner. Survival rate of the cells was assessed by the MTT assay. **(B)** ROS production in cells treated or untreated with theextract (100 μg/mL) and then irradiated by 100 J/cm^2^ UVA (+) or not (–). **(C)** Total GSH levels determined by DTNB assay. Results expressed as mean ± SD of three assays. Significant ^∗^*p* < 0.01; ^∗∗^*p* < 0.001 compared to untreated control. Analysis performed by two-way ANOVA followed by Bonferroni’s multiple comparisons test. **(D)** Immunoblotting bands of the oxidative stress activated protein, p38. An equal amount (100 μg) of total lysate from each sample was resolved by SDS-PAGE with GAPDH as a control.

### Hepatoprotective Activities

In order to validate the *in vitro* and cell culture results, we tested the antioxidant activity of the extract *in vivo.* Thus, the preventive action of the extract against the intoxication of CCl_4_ in rats was determined. CCl_4_ administration elevated all markers for liver damage. When the rats were treated with the extract prior CCl_4_ injection, protective activities were observed in all liver parameters. The extract (200 mg/kg b.w.) significantly reduced the elevated levels of ALT, AST, TB, TC, and TG, comparable to activities of the standard lignin from *Silybum marianum*, silymarin, **Figure 3**. Also, CCl_4_ injection significantly decreased the levels of GSH and SOD and increased MDA level in liver tissue homogenates. The extract markedly restored their levels to the normal control levels except for MDA, **Figure 4**. The hepatoprotection through the leaf extract was then further evidenced using a histopathologic study. The extract protected the liver against the deleterious effect of CCl_4_, **Figure 5**.

**FIGURE 3:** Hepatoprotection through a methanol extract of *S. aqueum* leaves in a rat model of acute CCl_4_ intoxication. **(A)** Alanine aminotransferase (ALT) activity; **(B)** Aspartate aminotransferase (AST); **(C)** Total bilirubin (TB); **(D)** Total cholesterol (TC); **(E)** Triglycerides (TG). Results are shown as means ± SD, *n* = 6, by one-way ANOVA followed by Tukey *post hoc* test. ^a^Statistically significant from the corresponding control at *p* < 0.05, ^b^Statistically significant from CCl_4_-treated group at *p* < 0.05.

**FIGURE 4:** Influence of a methanol extract of *S. aqueum* leaves on antioxidative enzyme activities in rats with acute CCl_4_ intoxication. **(A)** Liver glutathione (GSH); **(B)** Lipid peroxidation and generation of malondialdehyde (MDA); **(C)** Superoxide dismutase (SOD). Results are shown as means ± SD, *n* = 6, by one-way ANOVA followed by Tukey *post hoc* test. ^a^Statistically significant from the corresponding control at *p* < 0.05, ^b^Statistically significant from CCl_4_-treated group at *p* < 0.05.

**FIGURE 5:** Hepatoprotective potential of *S. aqueum* leaf extract on liver pathology after CCl_4_ treatment in rats, stained by hematoxylin-eosin. **(A)** Liver of normal control rat with normal hepatic architecture, hepatocyte structure and central vein. **(B)** Liver afterCCl_4_ intoxication with severe changes including dilated central vein with central hepatocellular necrosis (arrows) and congested portal triad. **(C)** Liver of a rat treated with silymarin prior to CCl_4_administration; only scattered cytoplasmic vacuolization (arrows) were detected. **(D)** Liver of a rat treated with the extract (200 mg/kg, b.w.) prior to CCl_4_ injection showing scattered cytoplasmic vacuolization (arrows).

### Anti-inflammatory Activities

Besides the antioxidant and hepatoprotective activity of theextract, we investigated its anti-inflammatory activity. In particular, we examined the ability of the extract to inhibit lipoxygenase (LOX) and cyclooxygenases (COX1/2). Interestingly, the extract inhibited LOX stronger than zileuton, the reference LOX inhibitor, as reported in **Table 3**. Additionally, the extract was able to inhibit both COX-1 and COX-2 *in vitro.* Moreover, the extract exhibited a SI value of 59.3, indicating higher selectivity toward COX-2 compared to COX-1. Noteworthy, the extract showed a higher COX-2 selectivity than that of indomethacin and diclofenac, but lower than that of celecoxib, as reported in **Table 3**.

**Table 3:** Inhibition activities of the extract on LOX, COX-1, and COX-2 enzymes.

	IC_50_ (μg/mL)	IC_50_ (μg/mL)	
Treatment	LOX	COX-1	COX-2	SI
*S. aqueum* extract	2.54 ± 0.19	7.11 ± 0.43	0.12 ± 0.005	59.3
Celecoxib	-	15.1 ± 0.72	0.049 ± 0.002	308.2
Diclofenac	2.11 ± 0.14	3.8 ± 0.17	0.84 ± 0.04	4.5
Indomethacin	-	0.041 ± 0.001	0.51 ± 0.02	0.08
Zileuton	3.51 ± 0.21	-	-	-

*SI is COX selectivity index which is defined as IC_50_ (COX-1)/IC_50_ (COX-2).*

In another experiment, we studied if the extract could counteract membrane disturbance in red blood cells (RBCs). At 1 mg/mL, the extract reduced the extent of RBCs lysis upon incubation with hypotonic buffer solution. Aspirin and diclofenac were used as reference drugs (**Table 4**).

**Table 4:** Effects of the extract, aspirin, and diclofenac on hemolysis of human erythrocyte membranes caused by hypotonic buffer.

Treatment	Concentration (μg/mL)	Hemolysis inhibition (%)
*S. aqueum* extract	1000	35.84 ± 0.93
Aspirin	100	68.32 ± 0.73
Diclofenac	100	81.63 ± 1.2

*Data is presented as mean ± SEM of three different experiments.*

We also explored the *in vivo* anti-inflammatory properties of the extract using the well characterized model, carrageenan-induced paw edema (Winter et al., 1962; Zhang et al., 2008). Rats pre-treated with the extract (300 mg/kg, p.o.) 1 h before sub-planter carrageenan injection (1% suspension, 0.1 mL/rat) significantly attenuated carrageenan-induced paw edema and decreased the AUC_0-24_ value by14.15 %. The positive control, diclofenac, decreased AUC_0-24_ value by 38.2%, as reported in **Figure 6**. The control group was set to 100%.

**FIGURE 6:** Anti-inflammatory activities of *S. aqueum* leaf extract. **(A)** Effect of 1 h prior administration of *S. aqueum* (300 mg/kg, p.o.) or diclofenac (10 mg/kg, p.o.) on carrageenan (1% suspension, 0.1 ml/rat) induced-hind paw edema in rats. Edema thickness (mm) was measured before and then hourly for 6 h and at 24 h after carrageenan injection. Data represents the AUC_0-24_ and are expressed as mean ± SEM (*n* = 5–7). **(B)** Effect of carrageenan (500 μg, i.p.) on leukocytes migration into the peritoneal cavity (total number × 10^6^) with or without 1 h prior treatment with the extract (300 mg/kg, p.o.) or diclofenac (10 mg/kg, p.o.). Data are expressed as mean. ± SEM (*n* = 5–7). ^∗^*p* < 0.01 vs. control values; ^#^*p* < 0.05 vs. carrageenan.

Carrageenan (500 μg/cavity, i.p., 0.1 mL) induced a significant leukocyte migration in the peritoneal cavity of mice (7.6 ± 1.2 × 10^6^ leukocytes/mL). Animals were pretreated with the extract (300 mg/kg, p.o.) 1 h prior carrageenan challenge; this significantly reduced leukocyte numbers by 50% when compared to vehicle-treated mice, (*p* < 0.05), as reported in **Figure 6B**. Similar activities were observed by a standard anti-inflammatory compound, diclofenac (10 mg/kg, p.o.).

### Antinociceptive and Analgesic Activities

In addition to the aforementioned activities, we researched the antinociceptive and analgesic activities of the leaf extract *in vivo* against acetic acid-induced writhing. As shown in **Figure 7A**, oral pre-treatment with the extract (300 mg/kg) almost abolished (96% reduction) the writhes induced by acetic acid in mice when given 1 h earlier (*p* < 0.001) compared to control. Diclofenac, a reference analgesic drug, achieved 65% reduction of the control writhes, (*p* < 0.001). These activities were also confirmed using hot plate test in mice where animals pre-treated with the extract (300 mg/kg, p.o.) prolonged the response latency when measured at 1, 2, 3, and 4 h after administration. This effect was significant at 1 and 2 h (14 ± 2.8 and 14.6 ± 2.5 s, respectively) post-treatment when compared to the control group (3.8 ± 0.5 and 4.2 ± 0.58 s, respectively). The standard reference drug, (nalbuphine, 10 mg/kg, i.p.), significantly increased response latency all tested time points with the maximum effect achieved at the 2 h (17.5 ± 3.37 s) (**Figure 7B**).

**FIGURE 7:** Antinociceptive activities of *S. aqueum* leaf extract. **(A)** Effect of *S. aqueum* extract (300 mg/kg, p.o.) or diclofenac (10 mg/kg, p.o.) on acetic acid-induced writhing (0.7%, 1 mL/100 g) in mice. **(B)** Hot plate response latency measured 1–4 h after vehicle, extract (300 mg/kg, p.o.) or nalbuphine (10 mg/kg, p.o.) administration in mice. Data is expressed as mean ± SEM (*n* = 5–7). ^∗^*p* < 0.001 vs. control values.

### *In Silico* Virtual Screening

*In silico* virtual screening studies were carried out on three crucial enzymes implicated in the occurrence and subsequent progression of inflammation namely, 5-lipoxygenase (5-LOX), cyclooxygenase-1 (COX-1) and cyclooxygenase-2 (COX-2). Most of the docked compounds showed certain stability within the active pockets of all tested enzymes except for samarangenin A and epicatechin-epigallocatechin-epigallocatechin gallate that failed to dock in both COX-1 and COX-2 owing to the relatively larger size of the molecules comparable to the active pockets of target enzymes (**Table 5**).

**Table 5:** Free binding energies (kcal/mol) of the identified compounds in 5-LOX, COX-1 and COX-2 active sites using molecular modeling experiments.

Compound	5-LOX		COX-1		COX-2	
	Rule- based ionization	pH –based ionization	Rule- based ionization	pH –based ionization	Rule- based ionization	pH –based ionization
NDGA (lead)	-44.49	-65.44	NT	NT	NT	NT
Diclofenac (lead)	-30.07	-34.64	-40.06	-40.72	-40.14	-40.74
epiGallocatechin gallate	-61.15	-56.22	-64.67	-66.33	-61.24	-67.13
Cryptostrobin	-31.58	-45.63	-40.80	-44.04	-39.60	-47.04
Europetin rhamnoside	-54.14	-58.23	-61.41	-63.90	-56.53	-66.52
Myricetin rhamnoside	-50.44	-61.19	-61.75	-57.07	-57.16	-67.74
Myrigalone B	-30.89	-31.62	-37.01	-37.83	-37.03	-41.87
Myrigalone G	-38.15	38.31	-43.49	-47.63	-49.87	-49.97
Samarangenin A	FD	58.70	FD	FD	FD	FD
Epicatechin-epigallocatechin-epigallocatechin gallate	-123.93	-123.62	FD	FD	FD	FD

*NT, not tested. FD, fail to dock.*

Among all the docked compounds, epicatechin-epigallocatechin-epigallocatechin gallate revealed the greatest stability with a pronounced highest fitting in the active site of 5-LOX displaying free binding energies of -123.62 and -123.93 kcal/mol, in the pH-based and rule-based ionization methods, respectively. In this virtue, it highly exceeds that of nordihydroguateric acid (NDGA), the potent well-known 5-LOX inhibitor that showed ΔG of -65.44 and -44.49 kcal/mol applying both previously mentioned methods, respectively. The apparent stability of epicatechin-epigallocatechin-epigallocatechin gallate in the active site of 5-LOX is strongly attributed to the formation of numerous firm hydrogen bonds with Ala 672, Asp 176, Gln557, Gln 363, Gln 609, Gly 174, Lys 173, Lys 409, Val 175, Val 671 and Thr 364 amino acid moieties in the active pocket in addition to a tight π-bond formation with Phe 177 as showed in the pH-based ionization method illustrated in **Figure 8**.

**FIGURE 8:** 2D and 3D binding mode of **(A)** epicatechin-epigallocatechin-epigallocatechin gallate in 5-LOX, **(B)** epigallocatechin gallate in COX-1, **(C)** myricetin rhamnoside in COX-2 active sites using molecular modeling experiments applying pH-based ionization method.

Regarding COX-1, (epi)-gallocatechin gallate revealed the highest fitting as manifested from the free binding energies, which are -66.33 and -64.67 kcal/mol in the pH and rule-based ionization methods, respectively. This firm stability in the active pockets is mainly due to the formation of six stable hydrogen bonds with Arg 120, Gln 192, Ile 517, Tyr 355, Trp 387 Ser 530 in addition to a π-π interaction and ionic bond with Arg 120 as revealed from the pH-based ionization method (**Figure 8**). Meanwhile, myricetin rhamnoside showed the highest fitting in COX-2 displaying free binding energies of -67.74 kcal/mol, in the pH-based ionization method with -57.16 kcal/mol in the rule-based ionization method. The tight fitting of myricetin rhamnoside in the active site of COX-2 could be explained in terms of the formation of four firm hydrogen bonds with Arg 106, Arg 499, Tyr 371 and Ser 333 amino acid residues existing at the active site in addition to the formation of a π-π bond with His 75 as illustrated from the pH-based ionization method (**Figure 8**). The presence of epicatechin-epigallocatechin-epigallocatechin gallate, (epi)-gallocatechin gallate and myricetin rhamnoside within the active pockets of 5-LOX, COX-1 and COX-2 were illustrated in **Figure 9**.

**FIGURE 9:** **(A)** Active pockets showing epicatechin-epigallocatechin-epigallocatechin gallate in 5-LOX, **(B)** (epi)-gallocatechin gallate in COX-1, **(C)** myricetin rhamnoside in COX-2.

However, the effect of ionization of different functional groups as well as amino acid moieties at the active site is well interpreted by the rule-based ionization method. This was reflected by the formation of an extra ionic bond between the phenolic hydroxyl groups that dissociate to form negatively charged phenolate ions in (epi)-gallocatechin gallate and positively charged amino groups as Arg 106 at COX-1 active site. Furthermore, an ionic bond was also observed between Arg 106 at COX-2 active site and the negatively charged phenolate ions in myricetin rhamnoside.

## Discussion

The present study profiled the phytoactive secondary metabolites and investigated the antioxidant, hepatoprotective, anti-inflammatory and analgesic activities of *S. aqueum* leaf extract in animal models and the underlying mechanisms. Utilizing LC-MS/MS, 87 compounds were tentatively identified, belonging to flavonoids, ellagitannins and proanthocyanidins. Promising antioxidant activities were obtained in all *in vitro* assays and in a cell-based model against the deleterious effects of UVA radiations. Also, the extract was able to counteract the deleterious effects of CCl_4_ in rats. These results are similar to previous findings from *Syzygium samarangense, Syzygium jambos* leaves and from other *Syzygium* species (Sobeh et al., 2018a,b).

We also assessed the anti-inflammatory activity of the extract *in vitro* by carrageenan-induced peritonitis, a suitable model of acute inflammation, in which vascular changes and production of inflammatory cytokines leading to leukocyte migration. We focused on the early increase in vascular permeability and neutrophil infiltration into peritoneum. The extract inhibited both cyclooxygenases, COX-1 and COX-2 with more inhibitory potential toward COX-2. Its effect on COX-2 was more potent than diclofenac but less than that of celecoxib. Furthermore, the extract inhibited lipooxygenase (LOX), thus suppressed leukotriene synthesis and inhibited RBC hemolysis.

In addition, the extract attenuated the carrageenan induced rat hind paw edema and inhibited carrageenan induced leukocyte migration. The effect of the extract was comparable but less potent than diclofenac. Also, the leaf extract demonstrated anti-inflammatory activity and produced comparable inhibition of leukocyte migration in comparison with diclofenac.

The response to pain stimuli in the hot plate test is attributed to the supraspinal reflex mediated by μ-opioid receptors (Le Bars et al., 2001). The antinociceptive activity is characterized by an increased tolerance to pain by the animal in contact with a heated plate. In the present study, animals pre-treated with the extract (300 mg/kg, p.o) significantly prolonged the response latency when measured at 1 and 2 h after administration. These results indicate that the extract also possessed central antinociceptive activity.

Altogether, the extract possesses solid antioxidant, hepatoprotective, anti-inflammatory, and pain-killing activities *in vivo*. These effects may be attributed to its flavonoid content, especially myricetin rhamnoside, quercetin glucosides, and epigallocatechin gallate. Flavonoids, among them quercetin, and tannins possess antioxidant, hepatoprotective and anti-inflammatory effects and play an important role in alleviating acute inflammation (Singh and Pandey, 1997). The anti-inflammatory effect of some flavonoids may be due to the significant inhibitory potential against many enzymes involved in inflammation such as phosphodiesterase, phospholipase A2, protein tyrosine kinases, and others. Furthermore, many flavonoids inhibit the major enzymes involved in the synthesis of prostaglandins and leukotrienes such as COX-1, COX-2 and LOX (Manthey et al., 2001). The extract is rich in polyphenols, which carry several reactive phenolic hydroxyl groups; they can partly dissociate to negatively charged phenolate ions. Polyphenols can form several hydrogen and ionic bonds with most proteins. As a consequence proteins complexed with polyphenols change their 3D structures and thus modulate their bioactivities (Wink, 2015; van Wyk and Wink, 2017). As this polyphenol-protein interaction is not specific, several proteins are involved, which would also explain the pleiotropic activities of our extract.

The results observed in the different *in vitro* and *in vivo* assays showed that *S. aqueum* offers good protection against oxidative stress, free radicals and oxidative stress related diseases. More detailed pharmacological assays are required before the findings can be translated into applications in humans.

## Ethics Statement

Hepatoprotective activities: The study protocol was approved by the Unit of Biomedical Ethics Research Committee, Faculty of Medicine, King Abdulaziz University, following the Institutional Animal Care and Use Committee guidelines. Anti-inflammatory and antinociceptive activities: The animal experiments were approved by the Ethical Committee of the Faculty of Pharmacy, Zagazig University for Animal Use and conducted following the guidelines of the US National Institutes of Health on animal care and use. Approved protocol for animal treatment is: P 9-12-2017, Faculty of Pharmacy, Zagazig University, Egypt.

## Author Contributions

MS performed the extraction, chemical characterization of the extract, the antioxidant activities *in vitro*, analyzed the data, wrote the paper, and conceived and designed the project. MM and SR designed and performed the anti-inflammatory and analgesic experiments and wrote the paper. GP and DM performed the antioxidant activities in keratinocytes and wrote this part. MA and FY performed the molecular modeling experiments and wrote this part. AE-S analyzed the data and revised the paper. AA-N performed the hepatoprotective activities and MW revised the paper, conceived and designed the project.

## Conflict of Interest Statement

The authors declare that the research was conducted in the absence of any commercial or financial relationships that could be construed as a potential conflict of interest. The reviewer SC and handling Editor declared their shared affiliation.

## Footnotes

1 www.pdb.org
